# The Significance of Shifts in Precipitation Patterns: Modelling the Impacts of Climate Change and Glacier Retreat on Extreme Flood Events in Denali National Park, Alaska

**DOI:** 10.1371/journal.pone.0074054

**Published:** 2013-09-02

**Authors:** Jill Crossman, Martyn N. Futter, Paul G. Whitehead

**Affiliations:** 1 Department of Chemistry, Trent University, Peterborough, Ontario, Canada; 2 School of Geography and the Environment, University of Oxford, Oxford, Oxfordshire, United Kingdom; 3 Department of Aquatic Science and Assessment, Swedish University of Agricultural Science, Uppsala, Sweden; University of Vigo, Spain

## Abstract

In glacier-fed systems climate change may have various effects over a range of time scales, including increasing river discharge, flood frequency and magnitude. This study uses a combination of empirical monitoring and modelling to project the impacts of climate change on the glacial-fed Middle Fork Toklat River, Denali National Park, Alaska. We use a regional calibration of the model HBV to account for a paucity of long term observed flow data, validating a local application using glacial mass balance data and summer flow records. Two Global Climate Models (HADCM3 and CGCM2) and two IPCC scenarios (A2 and B2) are used to ascertain potential changes in meteorological conditions, river discharge, flood frequency and flood magnitude. Using remote sensing methods this study refines existing estimates of glacial recession rates, finding that since 2000, rates have increased from 24m per year to 68.5m per year, with associated increases in ablation zone ice loss. GCM projections indicate that over the 21^st^ century these rates will increase still further, most extensively under the CGCM2 model, and A2 scenarios. Due to greater winter precipitation and ice and snow accumulation, glaciers release increasing meltwater quantities throughout the 21^st^ century. Despite increases in glacial melt, results indicate that it is predominantly precipitation that affects river discharge. Three of the four IPCC scenarios project increases in flood frequency and magnitude, events which were primarily associated with changing precipitation patterns, rather than extreme temperature increases or meltwater release. Results suggest that although increasing temperatures will significantly increase glacial melt and winter baseflow, meltwater alone does not pose a significant flood hazard to the Toklat River catchment. Projected changes in precipitation are the primary concern, both through changing snow volumes available for melt, and more directly through increasing catchment runoff.

## Introduction

Greenhouse gases, including CO_2_, alter the radiative balance of the atmosphere, increasing global temperatures, and altering precipitation patterns [1,2]. As these earth-system processes are intricately connected with river discharge, groundwater recharge and nutrient fluxes, these changes are likely to affect the quantity and quality of freshwater resources [3], with associated impacts upon biodiversity, and global and regional economics [4].

In systems containing large frozen water stores, such as those with headwater glaciers, climate change has the potential to have extreme and varied effects on a range of time scales [5]. It has been projected that increasing temperatures and altered precipitation patterns will initially lead to a general increase in rates of glacial recession and meltwater release [6], alter the timing and magnitude of soil saturation and runoff, lead to thinning of permafrost [7] and change lake levels and groundwater availability [8], thus affecting water quality [9,10]. This may be followed by eventual meltwater declines due to large depletions in glacier volume [5,11].

In glacial-fed catchments the annual flow regime is driven by a complex combination of processes including the build-up of snow during the winter, subsequent rates of snow- and glacial-melt during the summer, and rainfall contributions. Contributions of summer rainfall to runoff vary by catchment, partly depending on the size of the headwater glacier relative to the non-glaciated catchment area [12]. Due to the diversity and complexity of these catchments, there remains significant uncertainty as to the precise extent of the effects of climatic transformations at the local and regional level [13].

The ability to forecast the hydrological implications of future meteorological changes is becoming increasingly important under a rise in global population, and growing demands for freshwater. Hydrological forecasting is especially valuable in developing locally effective adaptation strategies for water supply, power generation, and flood mitigation [14]. Given the complexity of the individual catchment responses, hydrological models have been identified as the best available tool for obtaining this information, as they can incorporate projected changes in meteorological variables, glacial mass balance, and fluctuations in runoff and soil moisture [15,16]. When combined with a series of plausible hypothetical climate scenarios, these models can provide useful information on the implications of future climate change for catchment runoff [15,17–19].

There is, however, a general lack of long term data available for glacierised catchments [20], where efforts to establish permanent flow gauging stations are confounded by the remote nature of their locations, high energy braided rivers, and high rates of sediment transport. Thus, despite their large geographical extent and significant ecological and economical value, catchments fed by headwater glaciers are often neglected in monitoring programmes [21]. This presents challenges for hydrological studies, as many models require extensive observed datasets for model calibration and validation [22].

The glacier-fed Middle Fork Toklat (MFT) River, in Denali National Park Alaska, is one such remote glacierised catchment. It has been identified as being particularly vulnerable to climate change [23],, being fed by three small headwater glaciers, which have been estimated to be receding at around 24 meters per year [24]. It is a large braided system, subject to annual extreme summer flood events, which result in severe bank erosion, road damage, and occasional rock slides. The frequency and magnitude of these events are a concern both to tourist and mining industries, and in terms of ecological stability. Despite its vulnerability however, there are currently no long term flow records for the MFT River. Past attempts at in-stream monitoring have been confounded by the determination of only weak flow rating curves [21], attributed to high sedimentation loads and associated rapid channel migration.

In order to employ effective best management practices, a quantitative assessment of both current and future river discharge is required. This study therefore uses a combination of empirical monitoring and modelling to a) establish a strong flow rating curve and the first flow record for the MFT River Basin, b) calculate a long term glacial mass balance for the headwater glaciers, and c) project potential future changes in river discharge, with a focus on extreme flow events, under a series of future IPCC climate scenarios. By characterizing the catchment using a comprehensive hydrological model, based upon empirical measurements, the likely effects of various future climate scenarios can be assessed, including quantifying the influence that glacial recession will have upon the frequency and severity of flood events.

## Methods

### 1: Ethics Statement

The Middle Fork Toklat (MFT) River, a protected glacierised catchment within Denali National Park, is the focus of this study. All necessary permits were obtained for the described study, which complied with all relevant regulations. Permits were approved by the Denali National Park and Preserve National Park Service (permit number DENA-2011-SCI-0016).

### 2: Site Description

Temperature and precipitation are monitored hourly at the Park Entrance, approximately 60km from the study sites. Mean monthly temperature and precipitation in summer of 2011 were 9.2 °C and 37.0 mm, and in winter were -11.6 °C and 20.37 mm [25].

The MFT River catchment has an area of 131 km^2^, and is a north flowing tributary of the Yukon (63°31'2.47″N, 150°1'42.80″W). Three small headwater glaciers form a small portion of the catchment area, with a combined surface area of approximately 6 km^2^ (Figure 1), approximately 4.5% of the catchment land surface. In the valley bottom is an active braided floodplain, approximately 1,300 m wide at its greatest extent. It is formed by unconsolidated silts, sands and gravels which are glacial, fluvial and colluvial in origin [26].

**Figure 1:** Site map of the study catchment (63°31'2.47″N, 150°1'42.80″W), delineating major landuse types, and the location of the pressure transducers at the “flow gauging station”. Landcover data was obtained from the AK I&M Inventory Program (non-proprietary data), through the National Park Service data repository (http://nrdata.nps.gov/). Accessed 2013 August 6).

The geology and geomorphology of the MFT catchment are highly variable. Permafrost is found intermittently throughout, forming a shallow impermeable boundary in the upper soil horizon, and supporting several perched wetlands [27]. Extensively vegetated steep valley sides extend to the East and West, however vegetation is absent where gravitational reworking of rockfall debris has formed highly permeable debris fans and talus cones, due to the steep incline of the valley slopes. The western valley is comprised predominantly of sedimentary geological units, whereas the east comprises sedimentary, submarine basalt, and volcanic. A ridge of quartz-rich metamorphic rock runs through the north of the catchment. Snow packs are present at the summit of these valleys in May, and disperse rapidly throughout the spring [21].

Due to limited availability of long term flow data on the MFT, an adjacent catchment, the Teklanika, is included in this study. A 10 year flow record exists for this catchment [28], and its use facilitates a long-term regional calibration of the hydrological model. At 1317 km^2^ the Teklanika is much larger than the MFT catchment, however it is similar in many of its key hydrological and geomorphological characteristics (table 1). It is situated 12 km east of the MFT catchment, featuring a north-flowing river (63°27'4.674″N, 149°29'16.833″W). Similarly to the MFT, it is fed by a series of headwater glaciers which comprise only a small proportion of total land area (approximately 1.1%). Again the catchment features an active braided floodplain, comprised of glacial silts, colluvial sand and fluvial gravels [26]. Steep valley sides are densely vegetated by dwarf willow, legumes and grasses [29] interspersed with permeable debris fans and talus cones, mirroring those of the MFT catchment. The geology here is also very similar to that of the MFT, with the west comprised predominantly of sedimentary geological units, and the east of both sedimentary and volcanic [26]. A quartz rich metamorphic geological unit also runs through the north of the Teklanika.

**Table 1:** Comparison of catchment characteristics between Middle Fork Toklat and Teklanika.

Catchment	Toklat	Teklanika
Catchment Area (km^2^)	131	1317
% Glacial Cover	4.5	1.1
Geology of valley sides	Sedimentary, submarine basalt, volcanic, quartz-rich metamorphic	Sedimentary, volcanic, quartz-rich metamorphic
Floodplain Sediments	Glacial fluvial silts, sands and gravels	Glacial fluvial and colluvial silts, sands and gravels
Geomorphic Features	Glaciers, talus cones, perched wetlands, discontinuous permafrost	Glaciers, talus cones, perched wetlands, discontinuous permafrost
Vegetation	Dwarf willow, mosses, legumes and grasses	Dwarf willow, mosses, legumes and grasses

### 3: Flow Gauging

Flow depth and temperature were measured in the main MFT river channel for 31 days (20^th^ July to the 19^th^ August, 2011) using Minitroll In-Situ pressure transducers. The Minitroll is a self-contained datalogger, 18.3 mm in diameter, featuring a vented cable which automatically compensates for atmospheric changes and provides a more accurate reading relative to ambient atmospheric pressure. The study period was chosen to include the height of the glacial melt period which was expected to include flood events [21], and the onset of colder weather and associated low flow events. Measurements were taken continuously throughout the study period, with sensors scanned at 10 second intervals, from which 15 minute mean values were derived. Transducers were inserted into a 50 cm length of 4″ outer diameter PVC tubing, with 1 cm diameter holes drilled over basal 20 cm. The tubing was bolted to the upper half of a 1.5 m length of L bar, and the L-bar driven 1 m into the river bed, approximately one-quarter of the way across the river channel. The pressure transducer was secured, using steel cable, to the river bank.

Surface water velocities, channel cross sections and water depth were monitored at 50 cm intervals approximately every 3 days. To determine channel cross sections, measurements of stream channel dimensions, river depth and flow velocity (at 1/6 depth) were taken at a marked location. The cross sections were used in conjunction with the water velocity measurements to calculate channel discharge, calculated as Q = VA, where Q is discharge, V is velocity, and A is area.

A relationship was established between channel discharge and river depth, called a “stream rating equation”, using least squares regression. A significant rating equation enables river discharge calculations to be derived from in-situ flow depth measurements. The R^2^ value of the relationship between river depth and discharge in the Toklat River was 0.91, and the ration equation was:

Q = 117.53D^2^ -62.594D + 10.834

Where Q is discharge and D is river depth. Establishing rating equations in braided channels can be challenging, due to preferential lateral over vertical erosion [21]. To address this issue, the flow gauging site was carefully selected at a point where all flow from the MFT was constricted to a single channel. At the study site lateral erosion was restricted by a combination of rock fall debris and a series of channel reinforcement measures (steal gabions, and riprap). Channel width at this site was 6.6 m, with an average flow depth of 0.49 m. The maximum depth reached 1.57 m on 15^th^ August.

### 4: Long term glacial mass balance of the MFT River

In 2002, a longitudinal survey of the current centreline of one of the three headwater MFT glaciers was completed, allowing for general ice volume changes to be calculated when compared to photographic images taken in 1954 [24]. It was determined that the headwater glaciers were receding at an average rate of around 24m per year, with an average total volume loss of 6.88 X 10^6^m^3^ per year. These figures represent an average rate calculated over a 50 year period. It is important to establish rates of glacial recession at a higher temporal resolution, as it has been found that including these observed values, particularly of glacial mass balances, in hydrological model calibrations significantly improves internal model consistency and reduces uncertainties [20]. This therefore helps in establishing an accurate representation of the catchment hydrological dynamics.

Using a series of Landsat satellite images from the U.S. Geological Survey’s Earth Resources Observation and Science (EROS) Centre [30], a simple remote sensing analysis of glacial recession was performed between 1986 to 2009 (Figure 2). Only images of the highest quality (no pixel damage, and no cloud cover) and obtained during the height of summer (June to August) were used. Band 1 (wavelengths 0.45-0.52) of the electromagnetic spectrum was used for this study, as it is predominantly saturated over bright snow and ice, and contrasts markedly with surrounding areas of rocks and vegetation [31,32]. By using a standard summer-time period of data acquisition, the possibility of including snow cover in the analysis of glacial extent was minimised.

**Figure 2:** Remotely sensed images of headwater glaciers in the Middle Fork Toklat Catchment (63°23'46.67″N, 149°51'43.99″W), analysed using satellite data from 1986–2009, sourced from the U.S. Geological Survey’s Earth Resources Observation and Science (EROS) Centre of 1986-2009.

A succession of corrections was first applied to each image to account for differences in acquisition conditions (sun angle and intensity, satellite angle and satellite model). All images were converted from “model-specific radiance” (a common radiometric scale) to “at-sensor spectral radiance”, and then to “in-planetary albedo”, as described in [33–35]. This series of pre-processing analyses reduces inter-image variance and minimises errors during image comparison in relatively clear images [34,36].

On each satellite image, the termini of the three headwater glaciers were recorded, and the distance between marked points calculated. Recession rates of the ablation zone were then converted to glacial thickness, or “meters water eqv”, for use in glacial mass balance equations. By overlaying the terminus locations onto a digital elevation model from 2011, an estimate of depth of ablation zone loss was obtained (calculated as the elevation of the previous glacial terminus, minus the elevation of the new glacial terminus). Measurements were taken at marked increments around the terminus, and an average thickness calculated. This was multiplied by 0.9 (the average density of glacial ice [37,38]) to equate to meters of water equivalent (m water eqv). These rates of change in glacial thickness were then used to constrain the glacial mass balance within the HBV model. The DEM has a vertical resolution of 1 m, and recession rates exceeded this error bound in all analysis periods.

### 5: Calibration of HBV Glacial Mass Balance

The Nordic version of HBV (Hydrologiska Byråns Vattenbalansavdelningen) is a conceptual rainfall-runoff model, and incorporates a full glacial mass balance. HBV uses a series of observed values of precipitation, temperature and physical characteristics of a catchment. There are five main storage components in the model: snow, glacial ice, soil moisture, an upper runoff zone, and a lower runoff zone. The underlying physical processes, operating within and between these zones (such as snowmelt, glacial melt water residence times and evapotranspiration rates) are represented through simplified mathematical expressions [39]. The model is structured in a series of altitude intervals. During calibration, these expressions were adjusted via parameters within recommended ranges [40] to attain a “best fit” compared both with observed GMB/meltwater recession rates, and to observed river discharge records. A weather station at the Park Entrance was used to obtain the required 1965-2011 daily time series of precipitation and temperature.

Nordic HBV calculates hydrology in increments of altitude [40]. Snow accumulation occurs at an altitude level where precipitation is falling at a temperature lower than a specified threshold. This snow accumulates evenly to a specified storage amount, after which additional snowfall distribution may be lognormal. Snowmelt is calculated using a degree-day temperature index method. All meltwater is retained in the snow until the amount of liquid exceeds a specified fraction, after which meltwater may exit the snowpack. Below this threshold level, liquid water in the snow pack can re-freeze, but does so at a lower efficiency than meltwater. Each year, on a determined day, any snow which has accumulated above the storage accumulation threshold is converted to glacial ice. Glacial ice, when exposed (i.e. not covered by snow) melts in a similar way to, though at a greater rate than, snow.

The daily discharge values derived from the GMB (meltwater from snow and ice) are input into the soil moisture zone, a central part of the HBV model (Figure 3). This ultimately influences river discharge. Therefore, within glacierised catchments the glacial mass balance and related parameters are instrumental in constraining seasonal flow dynamics and projections of long-term climate change. It is therefore important to achieve an accurate calibration of these GMB parameters to prevent simulation of a) an unrealistic rate of glacial melt, b) to prevent inaccurate estimates of the relative contributions of glacial meltwater vs precipitation to river discharge [20].

**Figure 3:** A conceptual diagram of the HBV model, based on the description by Sælthun (39).

Glacial mass balance parameters, including the temperature at which precipitation falls as snow, the threshold snow accumulation levels (for ice conversion), and the rate of melt for exposed glacial ice were adjusted until the modelled average ablation zone water eqv (m) closely matched that of observed data for the same time period. This extensive calibration of the GMB improves the long-term accuracy of the HBV modelled glacial dynamics, and ensures a representative relationship between the GMB and meteorological data.

### 6: Calibration of HBV Hydrological model

The short duration of the available observed discharge data presents a challenge to calibration of MFT stream hydrology. Although flood events and low flow extremes were recorded during the study season, long term seasonal and annual trends were not. Much of this long-term uncertainty is reduced though the calibration of the HBV glacial mass balance to the remotely sensed glacial recession and GMB data [20]. With no observed winter flow data, however, there remains some uncertainty in inter-annual (seasonal) variation. To minimise this, regional flow dynamics of the area were first established through the calibration of HBV to a similar, proximal catchment (Teklanika), for which a 10 year daily flow record is available. This is a standard technique for “modelling flow in ungauged catchments” [41].

Catchment area and altitude interval data required for the calibration of HBV to the Teklanika catchment were derived from digital elevation models, using ArcGIS. Data requirements for potential evapotranspiration, temperature and rainfall were obtained from the meteorological station at the park entrance [25]; and surface runoff times, and groundwater residence times derived from the storm hydrograph. Additional expressions within HBV were adjusted within recommended ranges [42] to obtain a “best fit” compared with observed stream discharge. These included evapotranspiration constants, maximum soil water content, maximum infiltration capacity, percolation to different soil zones, and degree of draw up from groundwater. The calibrated HBV model was then applied to the MFT short-term dataset, and refined by adjusting parameters to account for differences in glacial extent, catchment area, altitude intervals, soil type, the presence of permafrost, and to include the calibrated MFT glacial mass balance.

No additional flow data was available for validation, therefore flow data from the Teklanika long term observed record was compared with a long term model simulation of the MFT catchment. This helped to assess whether the long term seasonal dynamics typical of glacial catchments in this region (summer discharge peaks and winter low flows sustained by groundwater) have been represented within the MFT model. As the Teklanika is a much larger catchment (table 1), the flow data was first reduced in magnitude by a factor of 2.6 (a factor calculated by comparing the average difference in magnitude between observed summer Toklat and Teklanika flows). It is possible that due to the difference in size, a slightly “flashier” response to meteorological impacts might be expected of the MFT. Therefore the flow data from the Teklanika catchment was used only for validation, and the MFT model was not adjusted to fit the long term Dataset As this is not true “observed data” for the MFT data, a direct assessment of model error cannot be made. The analysis does however demonstrate whether the model reflects the long-term hydrological dynamics typical of similar catchments in this area.

Maximum annual modelled discharge values (Qmax) were correlated with corresponding rainfall and temperature values, using Pearsons Correlation Coefficient, as a means of identifying dominant flood drivers. Due to non-normal distribution of data, all values were first transformed into z-scores.

### 7: Statistical Downscaling

Emission scenarios from two global climate models (GCMs), HADCM3 and CGCM2 were chosen to compare the degree of uncertainty in climate predictions. There are many different GCMs available, with demonstrable spatial variability in their accuracy. These particular models were chosen due to their high performance in arctic areas [43], and for the difference between their projections of changes in future rainfall [44], with CGCM2 giving much more conservative outputs. There are four scenarios in the IPCC fourth assessment report [45], each describing a hypothetical increase in population and technological advancement. The scenarios differ in their local, regional and global focus, particularly in the second half of the 21^st^ century, and represent different extremes of projected climate change. The A2 scenario demonstrates the highest GHG emissions, which progressively increase throughout the 21^st^ century, whereas the B2 scenario represents intermediate levels of GHG emissions, rising at a steady rate. These scenarios were chosen to represent both an extreme and a more conservative estimate of possible future changes.

The scenarios (A2 and B2) were downscaled using a Statistical Downscaling Model (SDSM4.2) [46], to provide regionally representative temperature and precipitation data for the MFT catchment. This technique uses regression methods that depend on the assumption that relationships can be established between the predictor variables at continental and local weather scales [47].

To calibrate the SDSM model, forty years (1961-2000) of baseline local observed meteorological measurements (predictands) were screened for statistical relationships and functions with regional National Centre for Environmental Prediction reanalysis data (NCEP predictors). These relationships were then applied to GCM predictors, under the A2 and B2 scenarios. This generates sets of local, long-term predictands (temperature and precipitation) for both HADCM3, and CGCM2 models. The precipitation series were downscaled following the procedure outlined by [46]. Precipitation downscaling is based on a conditional process, which assumes the existence of an intermediate process between regional forcing and local weather. An unconditional process, which assumed direct statistical links in the predictand-predictor model [46,48], was used to downscale temperature. Stepwise multiple regressions were used to calibrate the climate model. NCEP reanalysis data and the large scale HADCM3 and CGCM2 variables were made available by the Canadian Climate Impact Scenario (CCIS) and Data Access Integration (DAI) portal.

The accuracy of the downscaling results were analysed using a two-way ANOVA, to assess whether there was a statistical difference between the mean temperature (or precipitation) values of each scenario (NCEP, Observed and GCM) *within* each month (January to December), during the calibration period (1961-2000). Where significant differences were found between scenarios, post-hoc Tukey tests were conducted to establish the prominent time periods of divergence. An average (mean) of the A2 and B2 scenarios was used in the comparison with GCM scenarios, as all emission scenarios are standardised prior to the year 200, and so are statistically identical until after this date [49].

The downscaled temperature and precipitation data was then used as input data for the calibrated MFT River HBV model to generate a projected glacial mass balance and discharge data over 1965 to 2100. Percentage changes in temperature, precipitation and discharge were calculated between baseline (1980-2010) and future (2071-2100) periods. Values were calculated as averages (mean) over 30 year intervals, in order to represent the “climatic norm” of study periods. The frequency and magnitude of both baseline and future flood events were examined, using flow exceedance curves derived from the cumulative distribution function (CDF) of daily river discharge [50]. The magnitude of one in five year flood events (the 99.95^th^ percentile of the CDF, or those daily flows exceeding only 1/365x5 per cent of the data period) and of annual flood events (the 99.93^rd^ percentile, or those flows exceeding 1/365 per cent of the data period) was compared between baseline and future scenarios. Additionally, the number of peaks above the baseline flood event threshold values, for both 1 in 5 year, and annual flood events, were analysed over the future time series, to determine any future increase in frequency of flood events [51].

## Results

### 1: Glacial mass balance of the MFT River

Table 2 outlines the rates of glacial recession and thickness lost (m water equivalents) between 1986 and 2009. From 1986–2000, rates of recession calculated by this remote sensing method closely correspond with those calculated by [24] for the period 1954-2002, of 24m per year. Additional data presented here suggests that recession rates have more recently substantially increased, to around 68.5m per year by 2009.

**Table 2:** Historic rates of glacial recession and water loss as calculated from satellite data.

Year	Average Distance moved	Average rate of recession (per year)	Meters water eqv (ablation zone)
1987-1994	234.29	29.28	-3.59
1995-2000	148.46	24.74	-4.29
2001-2007	311.93	44.6	-6.14
2008-2009	163.23	68.55	-5.56

Loss of ice from within the ablation zone has also increased, from between -3/-4m in 1986-2000, to around -5/-6m per year in 2000-2009[24]. measured rates of loss on the East Fork Toklat Glacier (2km to the west of the MFT catchment) at -3m per year, and noted that rates would likely by marginally higher on the MFT Glaciers, due to their lower elevation. Calculations presented in table 2 correspond with these observations.

The HBV glacial mass balance, constrained to these recession rates, closely matched observed changes of glacial thickness in the ablation zone, with an R2 of 0.99 (Figure 4a). This high correlation between modelled and observed glacial mass balance gives strong confidence in the ability of HBV to represent the glacial dynamics of the MFT catchment (Figure 4b).

**Figure 4:** The water balance of Middle Fork Toklat headwater glaciers measured as equivalent meters of water a) in the ablation zone; comparing observed (satellite imagery analysis of glacial extent) and modelled (HBV glacial mass balance output) values, and b) analysing net glacial flux from the HBV model.

### 2: Hydrological dynamics of the MFT River

HBV was first applied to the Teklanika catchment, and captured both the monthly (Figure 5a) and seasonal flows well (Figure 5b), with R2 values of 0.83 and 0.95 respectively, Nash Sutcliffe coefficients of 0.81 and 0.97, and model error of 1.84% and 1.79%.

**Figure 5:** Comparison of observed and modelled discharge data in the Teklanika catchment a) on a monthly time scale, b) a 10 year average.

Upon applying the calibrated HBV model to the MFT short-term dataset, model accuracy of the summer 2011 events remained strong, with an R2 of 0.64 and N–S of 0.60 (Figure 6a). Model error over the summer calibration period was 21%. Upon validation using adjusted observed data from the Teklanika catchment, the model retained its representation of long term and seasonal flow dynamics, with a monthly R^2^ of 0.82 (Figure 6b) and inter-annual R^2^ flow values of 0.96. Although a quantitative assessment of model error is not possible for winter periods, due to the absence of MFT-derived empirical data during this time, the combination of a regional model calibration, combined with a locally constrained glacial mass balance and a short-term observed flow dataset, provide confidence that the HBV depiction of the MFT catchment is representative of reality. This study focuses upon summer periods, as this is both the period of interest concerning extreme flow events, and the period for which model error can be directly derived.

**Figure 6:** Comparison of observed and modelled discharge data in the Toklat catchment a) on a daily time scale, b) a monthly time scale.

The maximum annual discharge values are significantly positively correlated with precipitation (p = 0.03) (Figure 7a), with the majority of annual maximum discharge events corresponding with maximum annual rainfall amounts. Temperature values are weakly, though not significantly, correlated with high flows, and only where the two most extreme flood events are excluded from the analysis (Figure 7b). This suggests that these largest flood events are predominantly rainfall driven [5]. All flood events occur only in summer, when baseflow is elevated due to glacial meltwater contributions [52].

**Figure 7:** Exploratory analysis of the relationships between extreme flow events and a) precipitation, b) temperature.

### 3: Analysis of downscaled data: Comparisons of observed, NCEP and GCM

The two-way ANOVA demonstrates that mean monthly temperature and mean monthly precipitation simulated by NCEP data are not significantly different from observed temperature data throughout the 1961-2000 calibration period (p>0.01) (Figure 8a,b, table 3).

**Figure 8:** Comparison between observed, NCEP and Global Climate Model (GCM) meteorological data, between 1961 and 2000, demonstrating the representativeness of GCMs for a) temperature and b) precipitation.

**Table 3:** Two-way ANOVA performed on temperature and precipitation data (dependent variables) comparing mean values of scenarios (GCM, NCEP and observed) within different months.

Scenario	**P-value to NCEP**	Difference	CI lower	CI upper	**P-value to Observed**	Difference	CI lower	CI upper	N	SE
NCEP precip	**NA**	NA	NA	NA	**0.8244**	0.0401	-0.079	0.1593	444	0.0401
NCEP temp	**NA**	NA	NA	NA	**0.4473**	0.2712	-0.199	0.7412	444	0.1828
CGCM2 pptn	0.0112*	0.1427	0.0236	0.2618	0.001*	0.1829	0.0637	0.302	444	0.0463
CGCM2 temp	**0.999**	0.0263	-0.444	0.496	**0.363**	0.2975	-0.173	0.767	444	0.183
HADCM3 pptn	**0.1747**	0.0945	-0.205	0.2135	**0.6457**	0.0542	-0.065	0.1734	444	0.0463
HADCM3 temp	0.0105*	0.5672	0.0973	1.0372	**0.368**	0.2960	-0.174	0.766	444	0.183

The two-way ANOVA also demonstrates that, with the exception of CGCM2 precipitation, average monthly means generated by the GCM datasets (both temperature and precipitation) are closely representative of the observed local Toklat climate during the calibration periods, with no significant difference from either NCEP data, or observed data; indeed in the majority of cases the GCM datasets were statistically similar to both datasets. The similarity between all scenarios during these calibration periods gives confidence in the accuracy of the downscaling techniques.

As CGCM2 precipitation data differed significantly both from NCEP and observed data, Post-hoc Tukey tests were conducted to determine the origin of these differences (table 4). Significant deviations between the mean monthly values of GCM precipitation and a) mean observed and b) mean NCEP values are found during only two months (July and August), where precipitation is over-estimated. The influence of this two-month baseline period of over-estimation on general results is minimised by the subsequent use of seasonal averages (summer and winter). The absolute difference in precipitation amounts to a mean summer over-estimation of only 0.5 mm, a difference which is not significantly different from either the NCEP or observed data at the seasonal scale (table 4). It was therefore not considered necessary to perform a bias correction on the downscaled climate series; however the possible implications of a slight summer over-estimation by the CGCM2 dataset are considered throughout the manuscript.

**Table 4:** Post-hoc Tukey tests from two-way ANOVA performed on precipitation data, comparing (Test A) mean values of scenarios within specific months, (Test B) mean values of scenarios within specific seasons.

scenario CGCM2	Time Period	**P-value to NCEP**	CI lower	CI upper	**P-value to Observed**	CI lower	CI upper	N	SE
Test A	Jan	**1**	-0.4715	0.8090	**0.943**	-0.2590	1.10215	37	0.11645
	Feb	**1**	-0.6626	0.6179	**1**	-0.6985	0.5821	37	0.11645
	Mar	**1**	-0.6394	0.6411	**1**	-0.5579	0.7226	37	0.11645
	Apr	**1**	-0.4225	0.8580	**1**	-0.4205	0.8600	37	0.11645
	May	**1**	-0.8038	0.4767	**1**	-0.6928	0.5877	37	0.11645
	June	**1**	-0.665	0.614	**0.99**	-0.3540	0.9265	37	0.11645
	July	0.024*	0.037	1.3142	0.00*	0.3595	1.64	37	0.11645
	August	0.001*	0.1821	1.4626	**0.380**	-0.1223	1.1582	37	0.11645
	Sept	**1**	-0.9095	0.3710	**1**	-0.9113	0.3692	37	0.11645
	Oct	**0.344**	-0.1144	1.1661	**0.708**	-0.1887	1.0918	37	0.11645
	Nov	**1**	-0.8729	0.4076	**1**	-0.8493	0.4312	37	0.11645
	Dec	**1**	-0.6231	0.6574	**1**	-0.7546	0.5258	37	0.11645
Test B	Winter	**0.835**	-0.1323	0.3253	**0.761**	-0.1212	0.3364	444	0.09485
	Summer	**0.244**	-0.0632	0.4781	**0.023**	0.0254	0.5668	444	0.09485

### 4: Climate simulations: future temperature and precipitation

Average annual temperature increased between the baseline period (1980-2010) and future (2070-2100) across all scenarios (table 5, Figure 9a). Temperatures increased to a greater extent in the CGCM2 model (an average annual 3.00 °C rise in CGCM2 compared to an average 1.02 °C rise in HADCM3), and were more extreme under the A2 scenario of both GCMs (Figure 9a). Changes in precipitation were much more variable throughout the 21^st^ century (Figure 9b), though average annual precipitation between the baseline and future periods did increase across all scenarios (table 5). It might have been expected that due to summer over-predictions of the CGCM2 model compared to NCEP data, CGCM2 would demonstrate the greatest annual increases in rainfall. It is however the HADCM3 model which projects the greatest annual rainfall increases; as CGCM3 proceeds with a more conservative estimate of future precipitation change this suggests that the slight baseline over-prediction of CGCM2 had little to no influence on model results. In the CGCM2 model, changes in precipitation of the A2 scenario were around double those predicted by the B2 scenario (table 5). Conversely in the HADCM3 model, the B2 scenario projects a greater degree of change than the A2 scenario.

**Table 5:** Annual changes in temperature and precipitation under two different GCMs and IPCC scenarios.

		HADCM3	HADCM3	CGCM2	CGCM2
		A2	B2	A2	B2
	Baseline	-2.62	-2.64	-2.85	3.14
Temperature	Future	-1.51	-1.72	0.50	-0.518
	Absolute Change	1.12	0.91	3.36	2.63
	Baseline	1.07	1.05	1.27	1.30
Precipitation	Future	1.27	1.33	1.48	1.39
	Absolute Change(mm)	0.20	0.28	0.21	0.09
	% change	18.7	26.71	16.32	6.78
	Baseline	6.56	6.05	8.75	9.01
Discharge	Future	7.44	8.35	11.29	10.21
	Absolute Change(m^3^/sec)	0.89	2.30	2.53	1.20
	% Change	13.53	38.04	28.96	13.27

**Figure 9:** Complete modelled time series of a) temperature and b) precipitation across both GCMs and IPCC scenarios.

Under the CGCM2 model, temperatures increase predominantly during the winter, by 4.01 °C and 3.38 °C (A2 and B3 respectively) whereas in the summer only 2.43 and 1.57°C of warming is experienced (table 6). Under HADCM3 roughly equal amounts of warming are experienced during summer and winter under the B2 scenario, however more warming is experienced during summer under the A2 scenario (1.31 °C). Forecasts from the CGCM2 model indicate small reductions in winter precipitation (of 2.1 and 3.41%, or 0.01 and 0.02 mm in A2 and B2 respectively) (table 6), whereas the HADCM3 model forecasts a rise during this time (of 58.66% and 24.17%, or 0.39 and 0.18 mm under A2 and B2 scenarios). Conversely, the GCCM2 model forecasts increases in precipitation during summer (of 24.66 and 11.55%, or 0.52 mm and 0.24 mm under A2 and B2 scenarios respectively), where in the A2 scenario of the HADCM3 model small decreases are projected, of 4.73%, or 0.08 mm. Under the B2 scenario of HADCM3 however, a rise in precipitation amounts of 28.49%, or 0.42 mm is projected, similar to those projected under the CGCM2 simulations. Again, summer percentage change in precipitation is greatest under the HADCM3 model.

**Table 6:** Seasonal changes in temperature and precipitation under different GCMs and IPCC scenarios (s = summer; w = winter).

				**HADCM3**				**CGCM2**		
			**S**	**S**	**W**	**W**	**S**	**S**	**W**	**W**
			A2	B2	A2	B2	A2	B2	A2	B2
	Baseline		8.05	8.05	-10.25	-10.27	8.63	8.70	-11.05	-11.06
Temp	Future		9.36	8.96	-9.27	-9.35	11.05	10.27	-7.03	-8.22
	absolute change		1.31	0.91	0.98	0.92	2.43	1.57	4.01	3.38
	Baseline		1.62	1.48	0.68	0.74	2.10	2.13	0.68	0.71
Precip	Future		1.54	1.90	1.07	0.92	2.62	2.37	0.67	0.69
	Absolute change (mm)		-0.08	0.42	0.40	0.18	0.52	0.25	-0.01	-0.02
	percentage Change		-4.73	28.49	58.66	24.17	24.66	11.55	-2.10	-3.41
	Baseline		15.37	14.07	0.26	0.32	20.28	20.94	0.51	0.49
Discharge	Future		17.38	19.51	0.34	0.37	25.94	23.71	0.82	0.56
	Absolute change (m^3^/sec)		2.01	5.45	0.08	0.05	5.65	2.77	0.31	0.07
	% change		13.09	38.71	32.19	16.74	27.86	13.21	60.12	15.02

### 5: Future changes in glacial mass balance and river discharge

Under both GCMs, glacial melt is projected to intensify over the 21^st^ century. Projections from GCMs are similar until the 2030s, after which estimates are more extreme under the CGCM2 model (Figure 10a, table 7). Under the CGCM2 model, the net loss of ice between the baseline and future periods is estimated at between 8.216 and 11.43 m, whereas under the HADCM3 model it ranges from only 2.41 to 3.04 m. Under both climate models glacial melt is projected to be more extreme under the A2 scenario, by 0.63 m in the HADCM3 model, and 3.27 m in the CGCM2 model.

**Figure 10:** Complete modelled time series of a) glacial mass balance and b) river discharge across both GCMs and IPCC scenarios.

**Table 7:** Comparison of future changes in glacial mass balance, between different GCMs and IPCC scenarios.

Glacial Mass Balance		HADCM3		CGCM2	
		A2	B2	A2	B2
Net balance 1980-2010	Baseline	0.74	1.27	0.50	0.89
Net balance 2070-2100	Future	-2.30	-1.14	-10.93	-7.27
Loss of ice (meters water eqv)	Absolute Change	-3.04	-2.41	-11.43	-8.16

Similarly, average annual discharge increased under both GCMs, and both IPCC scenarios (table 5, Figure 10b). The greatest rises in annual discharge were observed under the HADCM3 B2 scenario (38.04%, or 2.30 m^3^/sec), and the CGCM2 A2 scenario (28.96%, or 2.53 m^3^/sec). During winter, discharge increased to a greater extent under the A2 scenarios of both GCMs, by 60.12%, or 0.31 m^3^/sec (CGCM2) and 32.19%, or 0.08 m^3^/sec (HADCM3) (table 6). During summer, increases in discharge were greatest in HADCM3 in the B2 scenario (38.71%, or 5.45 m^3^/sec) and in the CGCM2 model in the A2 scenario (27.86%, or 5.65 m^3^/sec).

Using flow exceedance curves of summer discharge (Figure 11) it can be seen that in all GCMs, the percentage time that a given flow is exceeded increased in the future scenarios. There was an increase in the magnitude of 0.05% flow exceedance (or 1 in 5 year flood events) and 0.07% exceedance (or annual flow events) under all scenarios (excluding HADCM3 A2). Discharge of one-in-five year events increased by between 15 and 60 m^3^/sec, and of annual events increased by between 16 to 28 m^3^/sec (table 8). By using the values of these flood events for the baseline 1980-2010 period as baseline flood thresholds, future peaks above this threshold can be used to determine changes in flood frequency (e.g. the peaks above threshold analysis [51]). This analysis demonstrates that under all scenarios (except HADCM3 A2) by the period 2070-2100, there will be an increase in frequency of flood events by between 1.6 to 2 times (annual events) and between 1.7 to 2 times (1 in 5 year events). The greatest increase in number of flood events occurred under the HADCM3 B2 scenario.

**Figure 11:** Flow exceedance curves under baseline and future climate conditions, demonstrating changes in the percentage of time particular flows are exceeded.

## Discussion

### 1: Effects of future climate on glacial recession and catchment hydrology

Projected increases in temperature and precipitation between 1980–2010 and 2070-2100 within the MFT catchment will likely have important consequences for both the glacial mass balance and river discharge. In catchments with contributions from glaciers, snowfall and snowmelt, these altered patterns can have significant effects [53,54]. Precipitation previously falling as snow may begin to fall as rain, increasing runoff in winter months. In addition, the spring snowmelt period may be brought forward [53,55], melting existing snow and glacial ice stores. Increased rates of glacial recession and associated flood events are currently of great concern within the MFT catchment [24,56].

**Table 8:** Changes in flood magnitude and frequency between baseline (1980-2009) and future (2070-2099) periods.

		Annual flow exceedance (0.07%) (m^3^/sec)			1/5 year flow exceedance (0.05%) (m^3^/sec)		Increase in number of peaks)	Increase in number of peaks
	baseline	future	% change	baseline	future	% change	over 0.07% baseline threshold (POT	over 0.05% baseline threshold
CGCM2 A2	154.87	178.57	15.30	235.00	257.22	9.46	22	4
CGCM2 B2	163.36	180.1	10.24	233/48	254.84	9.14	19	5
HADCM3 A2	152.28	146.08	-4.07	230.57	209.15	-9.29	-5	-1
HADCM3 B2	138.78	167.29	30.54	245.71	259.54	5.63	32	6

Results are expressed for both annual flood events, and 1 in 5 year flood events.

Future projections under both GCMs indicate that the glaciers will continue to melt, and at a higher rate than under the current climate. By 2070-2100 the threshold between accumulation of glacial ice in winter, and melt in summer is permanently crossed, and more ice is lost than gained. Under the projections from the CGCM2 model, the extent of this threshold crossing is more extreme, and the melting of the MFT glaciers most extensive.

Glacial winter accumulation and summer melt are related to the extent and timing of changes in temperature and precipitation [57]. The less extreme future projected temperature increases, and higher projected winter precipitation increases depicted by the HADCM3 model correspond with a more conservative projection of future loss of glacial mass than under CGCM2. These future projections of winter climate favour accumulation of snow and glacial ice. Projections for this GCM are most conservative under the B2 IPCC scenario, where temperature increases are also lower in summer, reducing the amount of glacial melt. Similarly, under CGCM2, less mass is lost under scenario B2, corresponding with the lowest projected increases in temperature. A2 scenarios project the greatest loss in glacial mass.

The increased glacial meltwater contributions combined with the changing climate have implications for river discharge. One such effect is increasing winter baseflows, indirectly caused by greater summer meltwater contributions, where melting permafrost under warmer climate enlarges the depth of the active soil layer, and facilitates extra groundwater storage [58,59]. Thus increased meltwater released during summer may be slowly released as groundwater during the winter period. In addition, increases in winter temperatures and in precipitation may contribute to a greater proportion of precipitation falling as rain (leading to increased winter runoff), and an increase in snowmelt (earlier spring melt) within the catchment [15]. Under the A2 scenarios, the more significant glacial melt, and the greater rises in winter temperatures and precipitation correspond with greater increases in winter discharge under both GCMs.

These effects may also influence summer discharge, where scenarios which accumulate less snow and ice during winter have a lower volume readily available for melt during the summer period [12,15]. In the HADCM3 (B2) projection, greater winter precipitation and lower projected temperature increases may contribute to the projected extreme increase in summer discharge, accumulating large snow stores for subsequent melt. Significantly this scenario also demonstrates the highest increase in summer precipitation. Discharge may be additionally raised through an increase in summer baseflow due to glacial melt, though this contribution is low in this scenario. The HADCM3 A2 scenario demonstrates a 50% lower rise in discharge than B2, corresponding predominantly with a projection of reduced summer precipitation. This demonstrates the potential significance of precipitation in this catchment during summer. Similarly, although in the CGCM2 B2 summer scenario there was much less glacial ice and snow available than in the HADCM3 A2 scenario, the projections of future discharge are similar (13.21% under CGCM2 B2 and 13.09% under HADCM3 A2). The higher summer precipitation projected under the CGCM2 B2 scenario likely compensates for some of the discrepancy in ice/snow-melt availability, and suggests that increasing glacial meltwater during the summer is not the dominant driver of river discharge amounts.

Changes in the nature of extreme flow events are also highly significant, with three of the four GCM/IPCC scenario combinations projecting increases in flood frequency and magnitude. Under the HADCM3 A2 scenario, however, reductions in flooding are projected, despite a similar future average discharge to CGCM2 B2. This reduction projected only under the HADCM3 A2 scenario corresponds with the projected reduction in summer precipitation, further highlighting the importance of rainfall as a driving factor in this catchment. In support of this, scenario HADCM3 B2, projecting the largest increase in frequency of flood events, also projects the largest percentage increase in summer precipitation. It is likely that in summer, runoff from greater precipitation amounts, falling on top of a higher baseflow provided from a higher rate of glacial melt and from melting of winter snow-melt stores (originating from greater winter precipitation) will more frequently create conditions conducive to flooding. Similar results have been discussed elsewhere [12] concluding that although temperature variations may alter the timing of discharge events, it is precipitation that is the most important predictor in changes in discharge amounts.

### 2: Wider Implications

Significantly this research determined that in the Toklat Catchment it was not the scenarios projecting the greatest degree of warming, or the greatest amount of glacial melt, which lead to the highest annual changes in discharge, flood frequencies and flood magnitude. Here rainfall is a significant factor, and the greatest changes in hydrology are observed under a more temperature-conservative IPCC scenario (B2) which in fact projects the least warming (HADCM3). The MFT is clearly a dynamic catchment driven by complex interactions involving winter snow accumulation (interaction between winter warming and winter precipitation amounts), summer glacial melt (interaction between summer warming and winter snow accumulation), and summer precipitation amounts.

These findings correspond with studies conducted in the Himalayas [15] which similarly found that although maximum glacial melt occurred under high temperatures, maximum stream flow was related to a balance between both temperatures and precipitation factors. Research in California examining streams at a range of elevations, with varying degrees of snowmelt contributions [12], also determined that the influence of precipitation upon stream flow variability is much stronger than that of temperature. Importantly, these studies found that the dominance of the precipitation influence is strongly related to the extent of glacial (or snow) coverage. The implication is that for locales experiencing glacial recession, changes in precipitation will become a progressively more dominant influence on flood frequency and magnitude than changes in temperature.

### 3: Uncertainty

There are a large range of uncertainties inherent in using hydrological and global climate models, ranging from the choice of GCM and IPCC scenario, to the quality of calibration of the hydrological models used.

To facilitate an assessment of the degree of uncertainty resulting from the selection of global climate models and use of IPCC scenarios, two of each were selected for use in this study. Although there were large differences in projected changes in temperature and precipitation amounts, all GCMs and IPCC scenarios were in general agreement that the rate of glacial recession will increase, and that there would be rises in both seasonal and annual discharge. The majority of GCMs and scenarios also suggested a likely increase in flood magnitude and frequency.

A sensitivity analysis was conducted of the model HBV to ascertain which key parameters exert the greatest control over model behaviour. In order to reduce parameter uncertainty and minimise equifinality (where different sets of optimum parameter values may yield similar model performance) it is important to identify these key parameters, and to calibrate them to observed data wherever possible [60]. The model was run over a series of 5000 simulations, with the top performing 100 iterations classified as “behaviours”, and the remainder as “non-behaviours”. Performance was defined as the sum of Nash Sutcliffe, and Nash Sutcliffe of log-transformed values. Where behaviours are non-uniform (i.e. the parameter is performing ‘better’ and has a significant influence on model output) a significant Kolmogorov-Smirnov statistic is derived. Kolmogorov-Smirnov statistics were therefore calculated for the cumulative distribution functions (CDFs) for each parameter in the behavioural set. The parameters are ranked from most to least sensitive in table 9.

**Table 9:** The top 7 most sensitive parameters, as determined through a sensitivity analysis of the Nordic-HBV model applied to the Toklat River catchment.

Parameter	KS	Mean parameter value	Standard deviation
KUZ1**	0.36	0.62	0.09
TX**	2.5	-0.67	0.48
CE**	0.24	0.37	0.09
TGRAD (7) **	0.22	-0.52	0.17
PKORR*	0.21	0.64	0.11
TS*	0.18	1.79	1.00
TGRAD (6) *	0.18	-0.38	0.20

** significant at the 0.001 level * significant at the 0.01 level

The rate at which water is conveyed through the soil zone to the river (KUZ1) was a highly sensitive parameter. This is to be expected, as the upper zone is the main dynamical part of the Nordic HBV model [40], through which hydrological inputs from snowmelt, glacial melt and rainfall are routed. As it is difficult to derive observed values for this constant, knowledge of relative permeability of local soil types are used. Further applications of Nordic-HBV to catchments fed by headwater glaciers will help to refine this parameter to within a range of recommended values.

Parameters relating to rainfall were also highly significant – these include the evapotranspiration constant (CE) and the correction for precipitation at meteorological stations (PKORR). This sensitivity might be attributed to the observation in the MFT catchment that precipitation falling as rain was the dominant influence upon extreme flow events during summer months. To reduce uncertainty in these measurements, pan-evaporation measurements might be taken from the site, and local rain gauges installed.

Finally, the sensitivity of a series of thermal parameters reflects the influence that the timing of snowmelt, glacial melt and snow accumulation have upon river discharge. These parameters include the threshold temperature at which rain falls as snow (TX), the threshold temperature for no melt (TS), and the altitude/temperature gradient (TGRAD) (i.e. the rate at which the atmosphere cools for every 100m elevation gain, predominantly effective in July). Here uncertainty could be reduced by installing meteorological stations at 100m increments on the headwater glaciers, including snow accumulation monitors.

In summary, this model application highlights catchment sensitivity to precipitation, soil permeability and temperature, i.e. that increasing summer precipitation corresponding with higher baseflow (from a melting glacier and a deeper active soil layer) will result in higher and more frequent extreme flood events, and this knowledge might be used for future adaptive management planning. However, collection of additional observed data would help to refine initial projections, and to unravel the complex hydrological dynamics inherent in this system.

## Conclusion

All future projections under the GCMs explored in this study indicate that the small headwater glaciers of the MFT catchment will continue to melt throughout the 21^st^ century, and at a higher rate than under the current climate. Due to increased precipitation during winter and associated accumulation of ice and snow, however, the glaciers also continue to contribute increasing quantities of meltwater to streamflow.

During winter higher river discharges are found under the IPCC scenarios projecting the greatest extent of glacial melt. This is likely due to melting permafrost facilitating extra groundwater storage. During summer however precipitation has the dominant effect on river discharge, with greatest increases in rainfall corresponding with rising discharge, flood magnitude and flood frequency. Three of the four IPCC scenarios project increases in flood frequency and magnitude, and again these events are predominantly associated with precipitation, rather than temperature or glacial meltwater contributions.

Results from this study suggest that although increasing temperatures will significantly increase glacial melt and river baseflow, the meltwater in and of itself does not pose a hazard to the MFT catchment throughout the 21^st^ century. Projected changes in precipitation are however likely to significantly influence discharge and flood dynamics, by altering the quantity of snow available for melt, and the water contributing from direct runoff during summer.
